This article has been retracted.

# Research on Effective Strategies of College Physical Education Interactive Teaching Based on Machine Learning

**DOI:** 10.1155/2022/1843514

**Published:** 2022-04-14

**Authors:** Zhe Zhang, Yinghui Zhang

**Affiliations:** ^1^School of Department of Physical Education, Yongin University, Yongin, Republic of Korea; ^2^School of College of Economics and Management, Wuhan Sports University, Wuhan, China

## Abstract

To master physical education courses, you must master a complete set of skills and knowledge. Most teachers still adopt traditional teaching forms, teacher centered, which has a negative impact on students. Because learners only passively participate in activities, it reduces students' enthusiasm and focus to master skills. This study is aimed at comparing and contrasting the differences between modern interactive learning and traditional teaching strategies. We collect qualitative and quantitative results about the impact of these studies on students' communication skills and understanding of relevant topics. The form of the noninteractive learning strategies explored in this study is the teaching system. This is a commonly used method and is still used in some institutions. Its limitations have led to the modernization of the education sector, especially in sports. This modernization brings about other forms of physical education, being student centered and more interactive. This form of interaction promotes the connection between teachers and students and promotes the transmission of feedback and the continuous improvement and novelty of activity forms. The interactive approach used in this study is the brainstorming method. Research has found it to generate constructive ideas and ideas. The specific process includes case study and Q & A, which is intuitive and clear, and can enhance the comprehensive understanding of the theme. The modernization of physical education curriculum brings many benefits; some of which will be listed in this paper. This study is aimed at promoting more display of students' personality in modern physical education teaching with clear research conclusions. Let the students in the training interact with teachers and interact with the group, in the interaction to play their own greater initiative, enthusiasm. Let the relationship between students and teachers be more harmonious, and let the students' physical quality get better development.

## 1. Introduction

P.E. is an essential aspect of the maintenance of physical and mental well-being [1]. Research has also indicated that, to some extent, it also improves the psychosocial aspects of an individual [2]. It presents with numerous health benefits. Together with its role in maintaining body energy balance, it can also control and treat chronic noncommunicable diseases like overweight and obesity. It achieves this by maintaining the body mass index (BMI) [3]. Physical activity also proves to be an essential aspect of musculoskeletal, metabolism, cardiovascular system, and, generally, the body's development processes. Its benefits are inexhaustible. There is an essential association between physical activity and health [4]. Physical activities can effectively exercise students' sports skills, help students to develop the habit of participating in physical exercise, so that students can maintain a good mental state for a long time, and pave the way for students to complete their studies and go to the society to meet the intensive work [5]. It proves the importance of the P.E. curriculum in higher learning institutions, especially colleges.

Notwithstanding the numerous benefits of it, many institutions have not been able to expose their students to the full benefits of these processes. It is because of low-content delivery strategies. The mastery of P.E. principles and skills requires a highly effective modernized education system. It is where interactive teaching comes in.

The interactive teaching mode is a teaching mode that highlights the main status of students and emphasizes the peer interaction of the behavior and emotion between teachers and students. It has important exploration significance for physical education courses with physical practice as the main means. Through the interactive teaching mode, strengthen the interactive communication between teachers and students, so that students can achieve new teaching effects in thinking ability, knowledge understanding, and skills. Through the interaction between the two, the current physical education teaching mode and teaching environment can be continuously improved and innovated in the interaction and the traditional one-way communication teaching mode of surgical courses of physical education specialty can be transformed into the communication and interaction between teachers and students, realizing the purpose of improving the teaching quality.

Teaching is as much an art as it is a science. It requires skills from both fields to be fully optimized and bring the expected outcomes. A study conducted by [6] has indicated the importance of interactive teaching styles in the P.E. curriculum. Some of these benefits are

- It facilitates a student-centered model whereby the content delivery is not teacher based but learner based. It excluded the chances of boredom, which was realized in the traditional system
- It enhances the concentration of the students throughout the activity. It is student centered, which means that other parts of the neurological system are continuously being activated
- It increases motivation. Interactive processes are efficient. The bonding process excludes the inferiority complex. It is because it is not instructor centered
- It continues improvement. Due to constant feedback, there is the periodic introduction of other novelty activities, improving the general processes and improving the outcomes

In the above study, various study methods were employed; some of which were interactive and noninteractive. Students were randomly selected from the school as the primary and study respondents; the thirty respondents were then divided into two groups. To reduce the incidence of bias, a double-blind approach was employed in this study. Both the students and instructors had no prior knowledge that research was being conducted.  Table 1 indicates some of the interactive and noninteractive research methods.

Table 1 indicates some of the traditional methods employed in teaching P.E.  Table 2 shows the currently used modernized teaching methods employed in the P.E. curriculum in college institutions.

Thirty respondents were randomly divided into two groups. Each group of students is then exposed to interactive instructional strategies (ITS) or noninteractive teaching strategies (NTS). The results show that the concentration time is negatively correlated with NTS when compared with that of modern teaching strategies. The scatter plots in Figures 1 and 2 show the different relationships between interactive and noninteractive teaching methods.

In Figure 1, the above result indicates that concentration increases with time in interactive teaching strategies vis-a-vis in noninteractive teaching methods. This research directed our study.

## 2. Method

### 2.1. Direct Interactive Model (DIM)

This model entails five instructional phases, each synchronized to work harmoniously to achieve the expected outcomes [7]. These five phases of DIM are

- Orientation phase
- Presentation phase
- Structured practice phase
- Directed practice phase
- Independent practice phase

All these phases can be diagrammatically represented as per Figure 3. In the orientation phase, the students become conversant with the subject matters of the session. It is where expectations and objectives are set. In the presentation phase, the relevant skills and contents are enumerated and explained by the instructors [8]. This process can be conducted with the use of relevant examples and real-life situations. It is indisposable that the instructor discusses the new concepts' characteristics and contextualizes the new content for the students. In the structured practice phase, the teacher helps the students perform the new skills stepwise. In the guided practice phase, the students are allowed to practice on their own. This phase happens while the teacher is still in the vicinity. In the final phase, independent practice assumes that the students have gained full mastery of the concepts. The instructor is thus out of the vicinity in the course of students' practice. Studies have shown that employing this model has helped in cognition and skill mastery than any other model in the teaching of physical education [9]. Figure 3 shows the superiority of the direct interactive teaching mode adopted in PE teaching.

Figure 3 shows the analysis and comparison between independent practical teaching and other teaching modes, believing that independent practical teaching has advantages in different stages.

As mentioned, a variety of strategies can be used in physical education. The purpose of these strategies is to turn the goal into practice in the process of teacher-student interaction in physical education class. These strategies are the product of the environment or situation. When the chosen strategy meets the needs of the educational situation, the strategy is irreplaceable; in the expansion stage, the selected strategy needs to use specific parameters. [10]. Because teaching strategies can adapt to the diversity of learning in the teaching process and satisfy the learning intentions, it can prove that people do not play a dominant role in teaching strategies. For example, Table 2 shows the modern teaching methods adopted in the physical education courses in universities and the impact between different learning strategies and environments on teaching practice and student grades.

Lecturing, PowerPoints, and handouts are the traditional teaching methods widely used in physical education teaching in colleges and universities. It is where an entire curriculum is taught using either verbal or visual means. In lecturing, the instructors deliver periodic verbal communication to a large group of learners. PowerPoint presentations involve the use of slides or any other visual digital format to communicate the content. On the other hand, handouts involve the use of printed takeaway notes to pass the content from the teacher to the students. These traditional methods have a tone of drawbacks, especially in the P.E. curriculum. As shown in Figure 4, we show the traditional teaching model. One of the cons of these models is that it is instructor centered. This reduces the degree of participation and motivation for the learners. It also facilitated boredom as there is no interaction between the teacher and the students [11]. Due to these drawbacks, modernized interactive methods have been put in place to supplement these traditional methods. There is specialized learning, simulation, and active participation with interactive methods, which are all learner centered [12]. These modernized models come with student centeredness, which increases the degrees of participation and concentration capabilities for the students, as shown in Figure 5. Some of the commonly used modernized teaching strategies are discussed in the subsequent chapters of this paper. Figures 4 and 5 show the traditional and modern teaching models, respectively.

Figure 5 shows the traditional teaching mode in college teaching. The traditional teaching is mainly teacher-centered oral teaching. Most students are not active in class. In teaching, they do not pay attention to the cultivation of students' consciousness, which reduces students' learning enthusiasm.

Figure 5 shows that the modern teaching mode has been innovated on the traditional teaching mode. This mode is mainly student centered. In the nutrition of intelligent machine learning, it can stimulate students' learning interest and learning initiative, which is more conducive to the current teaching needs of colleges and universities.

### 2.2. Personalized Method

The modern teaching strategy (MTS) of “division and governance” is adopted. It is aimed at discovering the characteristics of each student and at improving them on this basis. It considers each student's best learning strategy based on their thinking and ability to concentrate. The description is specific, involving only one requirement at a time. Therefore, the main problem with this teaching method is that it requires extensive early preparation. Because teachers need to have a lot of all the information about their students, it can waste a lot of time and resources. In some cases, this may be impossible. IAU uses intelligent systems to implement ITS and has the advantage that it can build confidence, because teachers only focus on one student at a time and students can also learn at their own pace [13]. This determines that each student has mastered the subject at the end of the event to begin the next stage.

### 2.3. Direct Interactive Teaching

In the MTS, there is a two-way interaction between students and teachers. The teaching content will be adjusted based on the feedback that the teacher receives from the students accordingly. The interactive teaching approach contains three stages, each independently ensuring the overall outcome of the course. Interaction means that both students and teachers influence each other and one person's reaction affects the whole process [14]. Innovation is a result shown postinteraction, and student feedback can enable the introduction and improvement of teaching practice; on the other hand, interactive education requires continuous feedback and student participation through discussion. The advantages of the ITS include the following:

### 2.4. Create the Content of Interest

This process is determined by motivation, so students are highly focused as compared to the NTS. The study also found that the process awakens many parts of the nervous system and keeps students' active participation in sports for longer.

### 2.5. Continuous Improvement and Feedback

It is because students have more feedback in P.E. class, enabling teachers to add freshness in the teaching process. The disadvantage of this teaching process is that, in some cases, it takes a lot of time and resources.

### 2.6. Simulation Teaching Method (STM)

It is another common MTS in physical education courses, which contains real-world environments and virtual scenarios [15]. Video records are generally used to achieve this purpose. For example, in PE classes, videos are used to guide students to PE classes and videos are played as learners mimic the process and activities. We enrolled five students in this MTS before taking a PE class to test for efficiency, the STM was performed using high-resolution projected YouTube video, and students should remember the audio and video content involved in the video process. Some sports equipment is needed on P.E., and the video uses the same equipment. They knew these processes better in real PE class than those who did not watch the video, and it promoted the full participation of five people. The results are shown in Figure 2.

Figure 2 obviously shows that in the efficiency test of student MTS in simulation teaching, there are significant differences between students participating in video simulation and students not participating in video simulation and the results of student simulation are also positively correlated with the increase of participation.

Peer teaching method in MTS, learned students act as teachers in the real-world classroom. Thus, it is more driven by learners than the previous methods. The advantage of this teaching method is that students with poor learning can learn from their good peers, eliminating the inferiority complex that may occur from teachers when teaching [16].

We conducted a cross-sectional study with randomly selected respondents to test the efficiency of interactive teaching methods against traditional noninteractive methods. The respondents' use was then taken through some of the interactive methods enumerated in the preceding sections of this paper. We use Figure 6 to visually show the relationship between feedback and conceptual mastery in the interaction model. The control group in our case was composed of those exposed to only the traditional teaching strategies [17]. Results indicated a positive impact on both the instructors and the students. In the part of the instructors, there was the aspect of introducing novelty skills and procedures based on the constant students' feedback. Constructive feedback facilitated the innovative processes of the P.E. sessions. In the students' part, the activities were more engaging. The fact that the physical exercises were also student centered other than instructor centered, there was increased participation on the students' part.  Table 3 shows the results of the study conducted.

Figure 6 shows that interactive teaching is more conducive to the mastery of learning.

## 3. Conclusion

The present study is aimed at exploring the application of interactive pedagogy in physical education courses. We have enumerated and explained the pros and cons of traditional P.E. teaching models and enumerated some of the modernized interactive strategies and how they are essential in mastering the skills.

## Figures and Tables

**Figure 1:** Correlational presentation between the different teaching methods and concentration. Outcome of interactive vs. noninteractive teaching strategy.

**Figure 2:** Efficiency test under different modes compared.

**Figure 3:** Direct interactive teaching model employed in P.E.

**Figure 4:** Traditional teaching model.

**Figure 5:** Modern teaching model.

**Figure 6:** Relationship between feedback and mastery of concepts in the interactive model.

**Table 1:** Traditional non-interactive teaching strategies.

Strategy	Definition	Effect
Verbal lectures	An instructor-based teaching method where the teacher presents periodic verbal sessions	Low concentration capabilities
PowerPoint presentation	Slides are presented with little explanations	Low motivation to the students. It can also be exhausting with bulky slides
Written handouts	The instructor issues printed notes to the students as takeaway jobs	Only a few students can follow-up and read the teacher's content. Poor feedback from the learners

**Table 2:** Modernized interactive teaching methods.

	Teaching strategy	Context	Effect
1	Simulation method (S.M.)	Real-life situations and encounters are simulated in the course of the sessions	A high degree of concentration and facilitating observation
2	Peer teaching method	The peer directs the sessions under the instructors' supervision	Student driven, thus a high level of concentration
3	Learning contract method	Clear documentation of the procedures and activities is done before the actual P.E. session	Objective based, thus high-order accomplishments
4	Q and A sessions	Constructive questions are presented for which the students are to come up with an appropriate answer for each question	Enhances students' thinking capacity
5	Active method	Students learn by doing other than just observation	Enhances full understanding of the topic in question
6	Task-sheet method	Records of the activities and procedures are kept using task sheets	Students can improve their weaknesses from others' strengths
7	Cooperative method	Group discussions and participation	Enhances teamwork
8	Problem solving method	The learning process is conducted by finding solutions to real-world problems	Enhances students' problem solving
9	Individualized method	Every student is an independent entity with different sets of activities and procedures	Every student's need is catered for and improved

**Table 3:** Comparison of students' participation in different teaching modes.

	Positive	Negative
Traditional	X	✓
Modernized	✓	X

## Data Availability

The data underlying the results presented in the study are available within the manuscript.
